The article "Clinical Application of Augmented Reality in Computerized Skull Base Surgery" was retracted in 2023. Reasons: unreliable results or conclusions; concerns about the data; concerns about the peer review; concerns about the citations.

# Clinical Application of Augmented Reality in Computerized Skull Base Surgery

**DOI:** 10.1155/2022/1335820

**Published:** 2022-05-11

**Authors:** K. Kalaiarasan, Lavanya Prathap, M. Ayyadurai, P. Subhashini, T. Tamilselvi, T. Avudaiappan, I. Infant Raj, Samson Alemayehu Mamo, Amine Mezni

**Affiliations:** ^1^Department of Information Technology, M. Kumarasamy College of Engineering, Karur, India; ^2^Department of Anatomy, Saveetha Dental College and Hospital, Saveetha Institute of Medical and Technical Sciences, Chennai, Tamil Nadu 600077, India; ^3^SG, Institute of ECE, Saveetha School of Engineering, SIMATS, Chennai, Tamil Nadu 600077, India; ^4^Department of Computer Science and Engineering, J.N.N Institute of Engineering, Kannigaipair, Tamil Nadu 601102, India; ^5^Department of Computer Science and Engineering, Panimalar Institute of Technology, Varadarajapuram, Tamil Nadu 600123, India; ^6^Computer Science and Engineering, K. Ramakrishnan College of Technology, Trichy 621112, India; ^7^Department of Computer Science and Engineering, K. Ramakrishnan College of Engineering, Trichy, India; ^8^Department of Electrical and Computer Engineering, Faculty of Electrical and Biomedical Engineering, Institute of Technology, Hawassa University, Awasa, Ethiopia; ^9^Department of Chemistry, College of Science, Taif University, P.O. Box 11099, Taif 21944, Saudi Arabia

## Abstract

Cranial base tactics comprise the regulation of tiny and complicated structures in the domains of otology, rhinology, neurosurgery, and maxillofacial medical procedure. Basic nerves and veins are in the nearness of these buildings. Increased the truth is a coming innovation that may reform the cerebral basis approach by supplying vital physical and navigational facts brought together in a solitary presentation. In any case, the awareness and acknowledgment of prospective results of expanding reality frameworks in the cerebral base region are really poor. This article targets examining the handiness of expanded reality frameworks in cranial foundation medical procedures and emphasizes the obstacles that present innovation encounters and their prospective adjustments. A specialized perspective on distinct strategies used being produced of an improved realty framework is furthermore offered. The newest item offers an expansion in interest in expanded reality frameworks that may motivate more secure and practical procedures. In any case, a couple of concerns have to be cared to before that can be for the vast part fused into normal practice.

## 1. Introduction

Augmented reality (AR) has gained tremendous adoption over the past two decades, but its use in the workplace is still being developed and evaluated. AR is a natural environment in which certified products are augmented with PC-generated virtual information. These partner markers are available in a variety of designs including sight, hearing, touch, smell, and taste. Augmented reality systems can be divided into two types, considering the level of sensation present in a given environment. That is, visible (momentary) and semi-determined (hidden) (hidden). Spectacular augmented reality hints at a structure in which the client articulates a real-world environment and additional data are projected onto it. However, translucent AR suggests a system in which the client is somewhat limited by the authenticated climate and cannot receive proprioceptive information about the body directly. In the workplace, AR can essentially be transmitted through glasses, shows, loudspeakers, gloves, joysticks, or jointly controlled robots. AR was first introduced in the 1960s under the name of “Theatre of Engagement” and takes the form of overlapping a real room with modern items [1]. The initial structure was redirect and bookmaker aware. Various fields have shown remarkable interest in the idea that was started earlier. A new leap forward in this field has paved the way for creativity to be showcased in a neat space. AR allows professionals to interface additional data available before or within the company into truly discreet realms, further extending cut points and approaches, treatments, survivability, and safety. With standard imaging techniques such as conventional X-bar, curvature tomography, attractive resonance imaging (X-beam), positron beam tomography (PET), and ultrasound (USA), or advanced imaging techniques such as practical X-beam (fMRI), experts can image Get, diagnose disease faster, and plan your workouts ahead of time in the smokehouse. The end goal is to continue using these structures. Today, standard CT channel, X-beam, ultrasound, and cone-bar CT (CBCT) can be used indoors without requiring a single moment to acquire small field images [2].

The article "Clinical Application of Augmented Reality in Computerized Skull Base Surgery" was retracted in 2023. Reasons: unreliable results or conclusions; concerns about the data; concerns about the peer review; concerns about the citations.

All image steering coordinate systems adhere to three basic principles: obstacles, bearings, and orientations [3]. (i) Constraints describe the work to be improved, such as development, actual plan, ulcer, or incomprehensible body (e.g., tool or insert) (e.g., tool or insert), and identify where the goal should be achieved. (ii) Orientation indicates the relationship between the patient areas with respect to the prudent instrument. (c) Pathways represent the most common methods of guiding a careful device to the best operation such as tissue resection, tissue fixation, fluid filling, or insertion of an insert.

Experts have approved imaging intercession procedure to remove visceral perversion that weakens the impact of standard imaging schemes such as endoscopes and microscopes. Image-based moderators have been shown to outperform standard strategies for both dominant outcomes and less disturbance [4]. Critical devices such as tactile analysis devices, remote-controlled computer controllers, and redesigned graphic shows are being manufactured to further push the limits of coordinated images [3, 5].

The most important benefit of AR in clinical interactions is the ability to view plans and recover hidden data without changing the mindfulness cycle. AR has been used for mindful organization, internal visualization, and deliberate pathway and target structure control [4, 6, 7]. In a general methodology, it would certainly be useful to indicate the base composition, infection, and risk locations. AR can also work with ambiguous methodologies, allowing experts to describe anatomy without disclosing it [8–10]. The major benefit of AR-based methodologies over traditional image matching strategies is the significant improvement in design ergonomics. With AR, everything is open from a single point of view, eliminating the need for experts to switch between error-free tactile structures (Figure 1). An important part of the distribution of the open AR structures recorded in hard copies is the hard [11–13], neurological [14–16], pancreatic, and hepatobiliary [17, 18] work. This is often due to the fact that this kind of clinical activity inhibits unimaginably limited organ development and transformation. (For the nuances of the gigantic augmented reality applications and other questionable applications in the classroom, assuming it does not require too much effort, see the attached current assessment [19, 20].) This remains unchanged. The limitations of working space, versatility, and demands for high accuracy (usually 1-2 mm) coupled with direct impact on residential structures have prevented effective use of AR here.

This article constitutes several review articles on the level of explicit termination that gives interesting fact on the use of augmented reality in neurosurgery, otolaryngology, and maxillofacial surgery [21–24]. However, these ratings relate to the application and not the specific credits of the available systems. Each of the newly expressed discreet strengths addresses a huge set of real-world domains (nose, ears, neck, head, spine pieces), thoughtful play plans, and different course requests. Alternatively, in this review article, we discuss the apparent cranial space difficulties and clinical interactions, the ability of the PC to support the process, and the potential outcomes presented by AR to update processes in this area.

The article "Clinical Application of Augmented Reality in Computerized Skull Base Surgery" was retracted in 2023. Reasons: unreliable results or conclusions; concerns about the data; concerns about the peer review; concerns about the citations.

Clinical management of the base of the skull is one of the areas that have benefited most from improved imaging capabilities [25]. This area separates the psychiatric larynx from the midface and neck. It provides an area for a huge number of cranial nerves and wires with the required capacity (Figure 2). Several material organs, such as the nasal cavity, ear, and eyeball, also surround the base of the skull. Therefore, it is very important to carefully understand the relationship between rigid structures and delicate tissues [26, 27]. Surgery at the base of the skull usually involves implanting, joining, shaping, or displacing parts of the skeleton to restore style and normal frame of life [3].

The base of the main skull is sometimes accessed through the nasal cavity using an inflexible endoscope inserted through the nostrils. A watchful view is displayed on the screen in front of the wizard. Research in this field includes accurate information on actual resting places according to 2D images and endoscopy headers and major limitations of 3D courses. In case of doubt, actual service stations will be changed or deleted due to previously used clinical drugs, contamination, or unnecessary waste [28]. Therefore, experts continue to use PC-assisted anterior cranial access as a reliable tool, despite a surprisingly long plan and experience [29]. The final screen shows a preoperative picture and the application site of the device. They constantly experience the reality presented by the system for judgment according to living design to support their decisions [29].

The flat bottom of the skull is often pulled closer through the stony bone containing the ear and important veins (carotid artery passageway, sinus sigmoid). This constituency requires extremely high-contrast tools and careful interaction. Sensory specialists break through the rock walls under meticulous reinforcement mechanisms, revealing actual development layer by layer and their progress into the cerebellar point and intracranial space of the pyramidal space [30]. However, the magnified focus provides a three-dimensional picture of the field, course, and bearing. Since the size and location of the actual part of the temporal bone vary greatly between individuals, it takes a long time for association and alignment [31]. As with nasal despondency, the destruction of achievement by disease, the organization of death, cerebrospinal fluid, and bone fragments can limit development. Rather, following the course screens while working with amplification equipment using anterior skull-based technology creates tremendous challenges. These two areas generally have a positive view. That is, it was developed from inflexible examples that are not flexible and not clear. This makes the PC-assisted course an accurate course for normally sensitive tissues.

The article "Clinical Application of Augmented Reality in Computerized Skull Base Surgery" was retracted in 2023. Reasons: unreliable results or conclusions; concerns about the data; concerns about the peer review; concerns about the citations.

A more accurate analysis and proactive planning have made management strategies in this area less cumbersome. Mortality and severity of interventions were significantly reduced [32]. Until the 90s of the last century, the usual system of control for the major base of the skull required a craniotomy with a direct view involving one or a pair of bony folds in the median plane [33]. Today, thanks to advance image-based planning, most strategies can be guided intranasally through the nostrils without visible scarring [34]. In general, a more precise method has been developed for the short-lived bones and the equivalent cranial base including the posterior fossa, and in some contaminations, it was normal to use the autopsy procedure and the endoscope together [35]. PC assisted meticulous tissue and demonstrated remarkable effectiveness in complex skull-based procedures. The real resting place here can be lost or obscured by disease. It can be cumbersome and unsafe to simply rely on visual perception to accept goals and reject critical plans through access to key openings, but so far, the pre-planned data are regularly reviewed in the minds of experts, rather than in a planned interface. By assisting with a careful perspective and using preoperative imaging information, practitioners can link their consent (goals and plans to move away) with more accurate and unambiguous outcomes to support an ideal deliberate work methodology [5]. A regular and thorough AR plan is shown in Figure 2.

This article analyzes several strategies presented using AR methodologies in specific real-world areas (basal of the skull and clinical treatment) and describes the different cycles used to treat interesting difficulties in this area. This seemed to be a smarter strategy than a strategy based on prudent qualities. Typically, these outlines are not provided in writing.

In this computed review, we will describe the efforts of AR on modern neurocurrent structures and the application of AR to clinical treatment in noncritical compulsive cranial settings. Then, around this point, let us take a concrete view of essential augmented reality. Finally, we will explore and test various methods of AR management and future contact with AR progression before AR is widely accepted as clinical therapy at our headquarters.

## 2. Approaches

In this review, we used a combination of the terms such as augmented reality, coordinated imaging, search, and medical procedures using the base of the skull, ears, and nose to fake a computerized study of public review dated October 2021 in “PubMed” in terms of otolaryngology, nasal, cranio-maxillofacial, sinus, base cranial, nasal cavity, otolaryngology, transitional bone, head and neck, and practical neurosurgery. The Fundamental Mission generated 250 tests. It eliminated duplicates and moderated the legitimacy of the review. We linked 45 tests to reviews to review and cross-reference 4 valuable articles.

The article "Clinical Application of Augmented Reality in Computerized Skull Base Surgery" was retracted in 2023. Reasons: unreliable results or conclusions; concerns about the data; concerns about the peer review; concerns about the citations.

## 3. Neuronavigation

Neuronavigation constructs are primarily aimed at directional developmental resection in neurosurgery. The incredible unpredictability of neuroanatomy has made it imperative to create incredibly accurate connections between patients and various devices and devices. Modern neuronavigation structures show central, coronal, and sagittal perspectives on a patient's preoperative CT or MRI, regardless of the screen. In addition to preoperative photographs, the application areas of various instruments are traced and clearly marked on the real plane [36]. This provides professionals with accurate 3D information about various gadgets. Neuronavigation is considered a common non-skull-based (MIS) operation increasingly used to move instruments when locked for review [36–38]. This is well suited for this application, as careful areas typically contain solid structures, allowing for ideal planning of preset useful openings. Multiple forms of information can similarly overlap each other during surgery to provide additional information [39]. A significant disadvantage of the neuronavigation structure is that the information is only displayed on different axes, and the expert has to intelligently blend information from different aircraft to find information about the course. In addition, this information is not available forever and cannot be seen from the master's point of view, which usually leads to problems that lead to tension and reduced accuracy [40, 41]. These inconveniences are further exacerbated by the complex basic living structures of flooded areas. Combining AR progression with neural navigation structures can provide significant advantages over standard neural navigation, but these developments have not been widely incorporated into careful game planning. The ingenious strategies available for prudent applications will undoubtedly cover many of the augmented reality systems in this industry. Various investigations have suggested coordinated image-based process architecture for endoscopic cranial augmentation surgery that allows professionals to perform the technique at a lower mental cost. This was accomplished by the provision of virtual planning boundaries and the use of global optical positioning structures for heading data [27, 42, 43]. On the other hand, according to Citardi et al. electromagnetic structures were used to provide course information for preoperative computerized tomography images and continuous endoscopic images [4]. For the convenience of customers, the main structures such as storage of the optic nerve, carotid artery, and installation method have been further expanded. The benefits of AR-based neural navigation systems with respect to time and workload recording used were quantitatively investigated, and their effectiveness was evaluated as largely error-free [44, 45].

The article "Clinical Application of Augmented Reality in Computerized Skull Base Surgery" was retracted in 2023. Reasons: unreliable results or conclusions; concerns about the data; concerns about the peer review; concerns about the citations.

Obviously, the impact of augmented reality systems was far more exclusive to less experienced professionals. Such kind of systems can also be useful for teaching and preparing for causes. AR could replace neural navigation technology. Unambiguous AR constructs have been developed that either provide exploratory information about underlying cognitive sources or provide direct patient/possible perspectives (Figure 3) [6, 7, 46, 47]. In the same way, robotic rescue AR could finally replace conventional neural navigation systems [48].

## 4. Applications in Minimally Invasive Surgery

A variety of prudent options are available for your skull crafting strategy. The open clinical strategy is the most common option for incisions of the face and skull to obtain target structures. Although this structure is best suited for objective planning, it creates more tissue damage around the methodology and may include organ dissemination, frustration, pain, anxiety, and prolonged postoperative stay in the center [27]. Similarly, cutting operations must be performed carefully to avoid destroying the command structures that exist in the area. Recently, MIS or keyhole surgery has become a non-routine solution. MIS refers to communication in which an alarm device and an endoscope are delivered to a target structure through a tiny entry point in the skin or skull. Regardless of how this contradicts many of the negatives mentioned, the limited perspective, lack of tactile sensation, and uneven progression provided by endoscopy add additional complications. If you do not have a 3D image, you can revise your assessment for a real-world situation. Moreover, since there is no horizontal view of the tunnel for all intents and purposes, access to open the key may involve cuts along the bearing [49]. These obstacles are very powerful in cranial formation and clinical interactions because they modulate important vascular and neural processes in the field of forced work. These angles can affect the awakening time, comfort, and persistence of professionals and ultimately lead to poor outcomes in terms of attention and adequacy [27, 50]. As a result, tools that further magnify images, areas, and postures turn out to be surprisingly basic when ordinary life structures are blurred. Specialists who monitor for problems at the base of the skull pay attention to brightening and marking by applying a strengthening focus. However, endoscopes give a two-dimensional view of a limited field, impede movement, and render certain images (30, 70) to reduce error-free vision segments, as well as light spot sensitivity [51]. The path towards the image can be associated with both an enhanced focus and an endoscope. The junction of the reinforcing focus or endoscope tip next to the focusing tool can be logically traced in the preoperative picture due to infrared radiation or the use of these devices [52, 53]. These changes allowed MIS to function properly and safely. AR-based MIS strategies have been recognized as supportive, eliminating accurate outcomes, and reducing the time required to deliver treatment [45]. In otolaryngology, AR has been used for ear support through the tympanic membrane (through the tympanic membrane) and mechanical cochleostomy [6, 8, 48]. In the nonscientific and clinical management of the base of the skull, AR is used to destroy damaged nasal tissue and provide information on basic laying plans and navigation rules [4, 27, 43, 50, 54, 55]. AR-based nasal endoscopy structural model films are available for download (under CC BY License) as Supplemental File 1 [50] (with CC BY consent). In the cranio-maxillofacial methodology, AR is heavily used to reproduce the cheekbones, providing information about the secret plan of the actual branch, but with no hope of disclosure [56, 57]. Figures 3 and 4 discuss, independently of each other, unique exhaustive AR applications for standard and MIS cranial methods, and these structures are fast and messy in the areas involved. In many augmented reality-based applications, the immersive data from preused data are superimposed on the original endoscopic camera image. Fields outside the endoscopic field of view are hidden from experts. The collected pictures were adjusted for structural processes of the endoscopic sinuses and the base of the skull. This is a clinical cycle that provides a fairly long view of the area of concern (Figure 3) [27, 44]. The endoscopic image is shown in the center, and the projection outside the scope of the endoscope is shown as a virtual reproduction of the previously used computerized tomography data. Several conferences have investigated the use of AR in real work settings for clinical management of the base of the skull [42, 45, 47, 55, 58]. This increasing cycle indicates that after progression and sequencing, AR can be used much more frequently and in a wider range of alarm conditions.

The article "Clinical Application of Augmented Reality in Computerized Skull Base Surgery" was retracted in 2023. Reasons: unreliable results or conclusions; concerns about the data; concerns about the peer review; concerns about the citations.

## 5. Methodologies

Different mechanistic approaches to AR are available by region name, but these mechanisms must match and apply to the base of the cranial region, keeping ergonomics in mind and carefully addressing the need for accuracy, consistency, and well-being of that particular region. In the image-oriented procedure, it is very important to build a general three-dimensional device inside the studio as a reference method. This usually ends with monitoring equipment changing patients, devices, and various devices [59]. These devices should not be a distraction from current prudent methodologies. The main aspects that determine the selection of devices and calculations are the time of registration and the accuracy of the verification. Clinically, recordings of 5–10 min and accuracy of 1–2 mm are recognized as reasonable tremors of the base of the skull [50]. Traditional photographic path structures are currently not ready to directly view virtual data from an operational perspective, which in turn increases the healthcare provider's brainpower to correlate navigational information with an accurate perspective. This has the potential to increase attention and confusion. Most of the AR scaffolds show accuracies greater than 1–2 mm, making them unsuitable for skull-based methodologies. To accommodate the specific requirements of this meticulous cycle, various methodologies have been introduced for arguably recognizable skull-based techniques. Most designs used optical tracking or electromagnetic devices that required additional patient-specific reference edges and markers, as well as sophisticated fixtures. A fixed person's head is usually fixed to a clip attached to the tracker. Hardware (e.g., super-imaging devices), CV (e.g., new photo-processing computations with capacity and optical flow based on the following [60, 61]), AI (e.g., faster and more advanced high-tech neural tissue [60–62]), and mechanical technology are gradually combined into one structure, and the components help the meticulous space. The current reality of error-free design can be explored in the relevant subsection. Existing thoughtful AR machines incorporate prepared processes such as gadget alignment, primer insertion, development supervision, gadget identification and validation, and perceptual conspiracy. The declared framework changes for each of these methods, and the final subsection provides an evaluation.

### 5.1. Calibration

Coordination is one of the most essential systems in this kind of equipment. A strategy for combining all the great vehicles is to deliver results within reasonable limits. The basic rule is to use as a reference a generic verifiable item with a predefined scope. The various subsystems that combine image capture and display devices, navigation ideas, surveillance designs, and sophisticated fixtures must first be coordinated before they can be used.

The article "Clinical Application of Augmented Reality in Computerized Skull Base Surgery" was retracted in 2023. Reasons: unreliable results or conclusions; concerns about the data; concerns about the peer review; concerns about the citations.

Each supported computer requires a careful tuning strategy to ensure accuracy. For certain projects, coordination must be cultivated before each rigorous task (e.g., a design requiring individually striking alignment that is affected [47]), while for others the best quality is first used (e.g., when the camera is the most limitations of the design required calibrations [27, 63]) (e.g., limits of designs where camera alignment is most necessary [27, 63]).

Previous AR structures have used ISG point size indicators or observation to adjust aspect ratio devices [56, 58, 64]. The method consisted of registering the position by hovering the tip of the pointer over a unique marker. Later, similar to the structure, a neuronavigation-style guide star was used to set up tools such as magnifiers, endoscopes, and routing devices [47, 50]. These designs use smart or optical markers attached to rigid patient guides with predefined points to align the anomalous device with the heavy person. Different kinds of designs have been proposed for pairing these markers, such as a hard shell attached directly to the cranium using screws or scarves, an outline attached to a Mayfield staple attached to the shoe itself, or a shell attached to the inside of a veneer [56, 57, 65]. The most famous tuning system in the clinical field is the photometric alignment method [6, 42–44, 65]. It incorporates a view (including its own view element) of a setup object from which actual 3D calculations are precomputed to determine the camera's inner and outer boundaries [66]. The articles to be sorted can be either a checkerboard test or a flat matrix. Devices containing cameras can take focal lengths from two images from a digital camera and align them to match [67]. The marker outline method provides remarkable accuracy [45, 57]. However, the appearance of the device indicates complications of surgery and limits the versatility of the device. Metering adjustment eliminates the need for an external body and provides an easy-to-understand strategy [66]. In any case, when the imaging device is connected to the magnifier, the photometric alignment system is usually limited in its performance as it has a limited set of fine focus perceptions. Whichever methodology you use, you need to think seriously because the regulatory system covers the entire region. Failure to do so could seriously impair accuracy when people travel outside of their designated locations. The ideal case would be when sorting is not required. However, such a design that pays attention to the high care requirements of the skull (ergonomics, insurance, reliability) for our excellent positioning is unrealistic.

The article "Clinical Application of Augmented Reality in Computerized Skull Base Surgery" was retracted in 2023. Reasons: unreliable results or conclusions; concerns about the data; concerns about the peer review; concerns about the citations.

### 5.2. Registration

A key step in a prudent AR machine is registration. Registration creates associations between interesting gadgets and special effects and solidly homogenizes them into a single mechanism. Recruitment is usually described as a structure of change that includes variables of rotation, interpretation, and deviation. Inclusion can be described as device (pictured person, patient device), order (2D-3D, 3D- 3D), or degree (hardness, firmness) (resolute, fortitude). The kind of registration your AR platform requires depends on the gadget you use. Getting started is the most basic methodology in a carefully crafted augmented reality framework because any issues that occur within an hour of this procedure will propagate for the rest of the journey. The most commonly used recruitment techniques are based on point-and-shape-based approaches (Figures 5 and 6). Physical attractions can be used to build engagement with photography throughout the registration process [8, 27, 68]. Configuring point-by-point registrations is often fast and requires much less registration effort. After all, physical markers are tedious to check and adjust as they move when the procedure starts or are covered with liquid, blood, or special effects. Also, the physical markers at the base of the skull are not clear, which can make selection problematic. Also, this system is not robust as it is basically impossible to select similar tourist destinations. Recognizable sham markers in both preoperative material and intraoperative images can be a trading choice [6, 42, 44, 69]. It can be fixed to pores and skin, or to bones. However, it is important that these markers merge earlier than the preoperative output, which usually occurs days before a truly thorough medical procedure. Markers should be static in equivalent motion during treatment sessions that limit patient movement. Alternatively, the markers can be stored in a separate, non-bendable shell attached to the victim's skull or trim. In conventional skull-based strategies, it is common to apply a discreet Mayfield cranial clasp to remove prominent markers. For AR technology, an exceptional type of dental design and occlusal braces focused on the maxilla or mandible has been created [56, 57, 65, 70]. These fiducial edges can similarly store markers for patient lists and unique attachments. These housings can also cause problems when transporting professionals and using tools. A picture marker will also be attached to the jaw of a weakened person and used for registration [71]. Using these markers rather than focus improves accuracy because image objects are used rather than error-prone careful focus [72]. You can also use sharp physical markers to improve accuracy. Surface scanners have been used in medical surgery since the mid-2000s and are expected to replace fiducial markers as the preferred choice for enrollment. Bones, entire surfaces, or shapes created using markers can be used for input [4, 47]. These methods are based on comparable loops coupled to rising frames or repeated proximity point (ICP) rule sets [7, 43, 48, 50, 73]. These techniques are surprisingly accurate but slow as they require a large number of shallow tricks (typically 200–500). If floor inspection is not usually possible, a fiduciary mark may be a second option. On the other hand, a combination of absolute strategies based on points and absolute bases can be used first to manage a core set by applying predicted or physical attractions, and then, approaches and gender adjustments are used to improve enrollment and vice versa [65, 72]. The combination of point and shallow match contains the advantages of both procedures, so it appears to be a quality of performance, but is computationally appreciated. On the other hand, the least serious registration method from a computational point of view is to ensure that the optical splitting line of the movable magnifier is used correctly, although confusing [46]. Incredible precision is critical when manufacturing incrementally additional parts.

The article "Clinical Application of Augmented Reality in Computerized Skull Base Surgery" was retracted in 2023. Reasons: unreliable results or conclusions; concerns about the data; concerns about the peer review; concerns about the citations.

### 5.3. Motion Tracking

Once recorded, listening to music on the patient's movements or holding the device is a great way to keep a great device connected. Like the registration process, it creates a transformation to show the entitlements between the old and newer stages. A huge part of the design is electromagnetic and optical design [11, 27, 42, 43, 50, 55, 57, 58, 63–65, 74]. There are many factors to consider when choosing a GPS beacon: number of devices to be monitored, charge of refreshing image, length of working area, power, basic accuracy, type of interaction with element environment, and area of next marker (if required). An optical tracker is a work of art that identifies infrared light received from an affected person or a reflective marker connected to one of the various devices.

Albeit new designs had been set up that give specific sorts of benefits yet, inferable from high precision, optical age stays to be one of the most extreme regularly utilized constructions inside the cranial base area. Electromagnetic and optical global positioning frameworks need strong reference outlines that fuse novel markers. To forestall this issue, different types of CV-based techniques have been introduced to tune any general movements among patients and picture catch gear [6, 7, 9, 71, 73]. To build precision, picture or fiducial markers may likewise be embedded into the global positioning framework. The issue with picture based completely following strategies is that checking is eminently done in 2D, and frameworks, which are not inside the picture body and inside the current day timestep, are not thought about. Movement observing is one of the significant parts of an AR machine since the image revive cost enormously depend on it. Along these lines, an astonishing spotlight should be put on picking a performant tracker. Different methodologies that affect picture revive costs incorporate photograph delivering and objective/device identification. Put together at the articles included with respect to this notice [4–7, 27, 42–48, 55–57, 63, 69, 73, 74] and financially accessible trackers, clearly optical trackers have shown the top-notch accuracy through trademark point coordinating with procedures give an ergonomic other option, disregarding a slight think twice about accuracy. Further developed innovative and farsighted basically based methods should be delivered in explicit, with the goal for them to be generously broad around here.

The article "Clinical Application of Augmented Reality in Computerized Skull Base Surgery" was retracted in 2023. Reasons: unreliable results or conclusions; concerns about the data; concerns about the peer review; concerns about the citations.

### 5.4. Equipment Identification

With maximum AR structure, the result is a two-dimensional image that ends up lacking persuasiveness. Similarly, when using a MIS strategy, the actual site is not immediately clear. This increases the need for augmented reality devices to access all the sensitive equipment and deliver data to healthcare professionals with interpretable technology.

The image on the left is an endoscopic view of the tympanic layer, and the image on the right is an AR exit showing the segmented central ear structure. Potential targets of the central ear, discernible only through magnified truth, have been indicated by (a) hammers, (b) anvils, (c) oval spears, and (d) circular spears. A discriminative model has been proposed to distinguish gadgets to enable technicians to gather the specific responsibilities of a device in a three-dimensional global realm. As with subsequent developments, advanced designs used electromagnetic and mechanical verification devices corresponding to devices [4, 64, 75, 76]. In any case, its structure was miraculously completely changed to an optical test structure that could be considered as the current of the device gradually as follows [11, 27, 42, 43, 55, 65, 69, 74]. These wireframes are clearly accurate and can be seen in most workspaces today.

The article "Clinical Application of Augmented Reality in Computerized Skull Base Surgery" was retracted in 2023. Reasons: unreliable results or conclusions; concerns about the data; concerns about the peer review; concerns about the citations.

Replacement units by design have also been favorably presented [6, 9], which better depend on data from the camera. Typically, a three-dimensional position is determined by attaching a primary visible marker recognizable by the video corpus to the device. While this strategy does not require bulky bezels or explicit labels, the device must remain inside the camera body all over the journey. These designs are also restricted by the quantity of devices that can be continuously detected. Despite encouraging verification results, mainly based on photographs, infrared optical trackers are still the preferred design choice after first-class performance [26]. The procurement department records the use of a personalized user-friendly interface with careful preparation and route information. The most common technique is to guide the tip of the device in three planes of symmetry with preliminary measurements [4, 27, 45, 55, 58, 76]. However, as recently explained, it is generally ergonomic for technicians to work with gadgets. Alternatively, you can use an alternate image that shows the tricky device directly in the augmented reality view. The 3D position is displayed as text on the presentation screen to capture the required movement. In any case, it is not ergonomic [6]. On the other hand, gadgets can inherently be presented in a specific color depending on the variance between them and an objective design [4, 55, 58, 65]. New developments that display device information on 3D show screens or in advanced/computerized 3D settings can be very lucrative and can help address challenges for healthcare professionals.

### 5.5. Visualization Devices

We analyzed different strategies for recognizing the consequences of augmented reality, including traditional screens, the age of wearables, and viewing and projection gadgets created for clinical exercise. A few examples of augmented reality shows are shown in Figure 7. The best representation of the AR structures at the base of the skull is the plain neat display cases [8, 42, 48, 50, 55, 65, 74]. This trend is evident when using an endoscope and in cases where direct viewing is usually not possible, including MIS techniques. An important advantage of this method is that other general practitioners can find patients at similar times at work. Nevertheless, in front of acoustic system magnification instruments and open medical procedures, AR shows are not a direct operational vision and appear increasingly lower in neat areas and AR output, resulting in tedious comparisons and broadcasts. Unlike conventional presentation screens, tablets have been used in a variety of applications and software packages to reveal hidden anatomy, which does not need significant incisions in cranio-maxillofacial strategies [77]. However, they are not increasingly strong in the otolaryngeal and nasopharyngeal ligaments because they belong to small and problematic life systems and to the more surprising principles of precision. Undoubtedly, the orifices of the nose and outer ear are unpredictable chamber conditions with a fairly high height for their size. Likewise, the lens frame is small and deep, so it needs to be lightweight and amplified. Moreover, the precision necessary for such rigorous methods cannot be achieved with standard innovations. Another drawback of standard presentations is that they do not provide an indication of depth at this stage. To do this, you will need to do extra work to be able to attack cautious units and targets. To assist professionals, fully data-based literature materials are usually provided in store windows [6]. On the other hand, a 3D showcase can be used to offset the depth perception problem [78]. Virtual reality reduces the perceptibility of prudent sites, and it is very important to understand that from now on, eventually introducing computerized ones in complete prudent terms no longer seems ergonomic. When evaluated, the efficiency of the PC can also be supported if the virtual structures overlap exactly as they are primitive, as shown in [55]. Native video footage or vividly rendered discreet moods are all other methods used to naturally view structures in three-dimensional space and convey enhanced authenticity [7]. Each pixel behind the focus emits light in a specific way. Healthcare professionals best consider the location of the emitted weak beam that can be immediately projected to the healthcare provider. This will make the salient part of the subject stand out from the odd title, giving the impression of power. Surface-based transportation or quantity-by-quantity beam tracking is commonly used to create showcases. A half silver reflection in the AR structure is associated with the show, allowing the expert to see the image of the idea superimposed on the person in trouble. Vital video is a smart choice because it is simple and allows parallax motion in both xy and *z* directions. However, the introduction of improved data is impossible due to the helpless execution of the gadget. A head-snared show (HMD) is an always-on device that includes a tiny show in front of one (monocular) or each (binocular) eye. Some HMDs also capture pictures for viewing by clients. With care, the helmet cap can overlay PC-generated virtual objects throughout the movie. This can be done both electrically and partially through intelligent radiation. Tablet-like HMDs are primarily used in a limited number of cranial-based projects and are now primarily used within cranio-maxillofacial areas that do not include very sensitive areas. In a rather vivid environment, it is possible to impose secret physical frames and route information on the patient. Binocular HMDs are not fixed to have better performance than single HMDs. Considering the effect of three-dimensional effect while maintaining good shape with careful handling of the head base, it was concluded that the use of binocular HMD resulted in a normal 35% improvement in accuracy and time of each conditioner compared with the monoscopic inventive reasonable [63]. The development of the HMD now apparently did not affect the localization of the target. HMD helmets provide ergonomics, including direct sensitivity, as opposed to the perception of a neat visual display, but have been proven to aid inadvertent blindness, especially when traumatic situations occur [74]. Inattentive visual impairment suggests an inability to see completely visible but unexpected things inferred from reality exchanged with focused attention on other actions, events, or articles [79]. Stylishly styled HMDs have not been widely used in clinical practice. This is due to the variables involved. (b) Delays: delays in the introduction of real and virtual information cannot be passed without serious consequences in a prudent environment. (c) Projection: it is easier to start at the end with an alignment strategy that defines the change between 3D world orientations as 2D images. These changes may now be irrelevant when optically transparent HMDs give HMDs key regulatory obligations. HMD devices are bulky and clunky devices, and this view is an excuse that many professionals do not like wearing HMDs. These designs can also keep clinicians busy, so this innovation is used appropriately.

The article "Clinical Application of Augmented Reality in Computerized Skull Base Surgery" was retracted in 2023. Reasons: unreliable results or conclusions; concerns about the data; concerns about the peer review; concerns about the citations.

### 5.6. Experimental Validation

The base of the skull contains the smallest and most fragile anatomy in the human body, and for image-oriented frames to function, their accuracy must be less than 1–2 mm within the elements of the workspace environment [6, 8, 80]. The target accuracy of AR frames you can get for money is typically 1.5–2 mm. In any case, as a rule of thumb, mistakes exceed this level [81]. Most experts already believed that, without sub-millimeter accuracy, the AR framework would have no chance of gaining recognition from experts. However, recent studies have shown that defects smaller than 1 mm cannot be identified due to the practical limitations of biological systems and devices, reducing the error to one in most cases. 5–2 mm have been suggested as conceivable [80, 82]. Equipment created under normal working conditions is tested at the Ghost and Corpse Bone Research Center before being performed in clinical settings on living things and humans. To work with evaluation frameworks, in some cases, most of the generated spurious markers may be accustomed to using an evaluation approach [43, 50, 57]. On the other hand, internal or post hoc analysis or informative legacy GPS beacons can also be used to determine objective accuracy [11, 71]. It is emphasized that when used with caution, the effects may differ significantly from those in a research facility. Also, errors occur as the distance between the camera and target increases [65]. Because of the complex living systems and workspaces, it is generally unbiased to rate presentations fairly. Therefore, several tests in humans provide the most subjective assessments [46–48, 55, 64]. In fact, no survey provides results for various tests [6, 50, 65, 73]. It is very clear from this study that the accuracy almost decreases at 45% use as we move from the research center to the workshop. Various components mandate final accuracy and design evaluation. (a) Enrollment baseline error (FRE) shows differences between reference areas (usually used for registration) in preoperative pictures, and the comparison focuses on individuals burdened with configuring the gadget. (b) Focus limiting (FLE) real is the distance between the hypothesized and actual focus positions as a result of the contrast within the image with the individual secondary structures affected. PPE is independently nonuniform and anisotropic in value and orientation. It is generally risky to engage in immediate and consistent training by averaging the various constraints of the equivalence part. (c) Target registration error (TRE) represents the intraoperative distance between the actual target constraint area and its location within the patient's tissue structure. This usually stands out due to the impeccable precision of the machine. (d) Overlay error (OR) is the same as TRE, despite the fact that proficiency in the intersection of projected virtual ideas and related designs in body space is recognized. It is usually assumed to be the boundary point of the projection. (e) Tool usage error (TE) is the directional error in units of attention used to implement the context definition and method. Finally, mistakes made in the show (lack of selection, contrast, magnification, or unadapted field of view) can further affect the complete result.

All the above factors are key characteristics of AR machines and require evaluation. For AR innovations to be effective in skull-based methodologies, analysts must focus on 1 mm sub-defects for each of the standards. Figures 3 and 4 show the impact of the different kinds of error auditing used in each view. Decisions about the scope of the assessment depend on the substructure of life, the type of perception, the level of implantation and enrollment, and the observation framework used. However, it is a good idea to talk to your TRE regularly, as it combines odd questions into one and gives you an excellent instinct for the absolute correctness to be expected.

The article "Clinical Application of Augmented Reality in Computerized Skull Base Surgery" was retracted in 2023. Reasons: unreliable results or conclusions; concerns about the data; concerns about the peer review; concerns about the citations.

## 6. Discussion

In the form of the project, the experts used a photo-centric scheme. From rigorous symptom-based interventions to intraoperative imaging, routes, and easy-to-use assessments, image-based innovations have a fundamental role in expanding the impact of treatment. The clinical goal is to overcome the shortcomings of outdated strategies that can complicate intraoperative appraisement and lead to inadequate execution. AR time has brought an additional perspective to such a framework. The combination of augmented reality with clinical imaging and atomic therapy (for cancer readers) provides specific physical local finding and integration of pre- and intraoperative data in an ergonomic and environmentally friendly methodology. The basis of the AR machine at the base of the skull is the precise reality of a very dangerous scaffold with veins and major nerves to prevent unwanted situations from occurring. In AR devices, virtual tricks can be superimposed on the real world as an approach. (a) Annotated or advanced models assembled in a pre-planned strategy are projected onto the sophisticated film. (b) The real world of the discreet film is combined with the virtual image. Previous versions of augmented reality used standard sensors such as optical and electromagnetic devices to communicate with interesting devices and customize every movement. The first bundles in the late 90s used electromagnetic observation methods that relied entirely on sensors in the lobby to set up tasks and tools [58, 64]. The problem with this age is that the details of a beautiful home can interfere with the results of the device. Thus, in the 2000s, optical design gained prominence and replaced electromagnetic design as the primary choice for developers [11, 27, 42, 44, 55, 63, 65, 69, 73, 74]. Optical trackers are currently considered the newest sensors in the preventive space. Careful devices and obvious devices may also be recorded using mechanical hands, which do not include relief scores [43, 48, 58]. The advantage of using such a design is that it provides an unreasonably high level of accuracy essential for cranial techniques. Since it does not rely on image processing, you no longer need to look at the edge of the endoscope while inspecting the tracked object. However, these generic structures require explicit pointers and wrappers to follow the more cumbersome process of reconciliation of the past than using them. Some frameworks do not require adjustments until after each thorough processing, but require re-tuning regardless of whether they are used under various environmental factors. Likewise, these designs require more memory in the work area and are incredibly heavy and bulky, causing anxiety throughout the session [42, 73]. Besides, this global positioning framework is really nice. These shortcomings have led to yet another innovation in AR architecture (with little or no real verification system), which essentially requires a computer camera connected to a surprising PC. Reality limits the scope of vision-based computations to instruments and instruments outside the outline of the camera, as the space outside the scope of the endoscope remains a definite position in vision-based augmented reality technology. Another important test that is uniquely and intelligently entirely AR-based is the helpless precision achieved in the entire operation of these designs. As a result, the high accuracy requirements required conventional transducers inside the base of the skull. However, modern advances in visualization, innovation, and the PC herald something unique, insightful, concrete, creative, and intelligent that is entirely based on AR architecture. Initial calculations at this stage have not yielded accurate results (greater than 1 mm) [7, 46–48, 71, 73]. This is ideal as more successful vision-based fully augmented reality projects prepared with visual and attractive control structures emerge [6, 8]. A shift to a full AR-based unique and insightful is coming, but similar adjustments are required to establish corporate balance within the cranial region. In work involving a thorough study of the base of the skull, endoscopic methodology of the sinuses and base of the head have all the indications that AR is the main area of use. An ideal augmented reality device must meet exceptional requirements. A system that incorporates a focusing marker and device and adjustments (which must be done prior to actual skill) on the burdened person should be simple and trivial. Thorough procedures aimed at images tend to have less depth of belief. Additional depth signals should be advertised for safety. In many applications, the virtual 3D objects are superimposed on endoscopic images, and it is necessary to provide a 3D image to maintain parallax when changing the viewing position. To present the best possible performance of virtual data, close attention must be paid to the format of the meticulous AR structure. This can darken key designs or cause visual pain, which can degrade your online experience in the field. Also, virtual recordings are best requested at time intervals other than all methods [11, 83]. Inattentive visual impairments also occur when relying on AR frameworks. Visual clutter can be avoided by performing spatial dating between prominent structures and removing obstacles [83]. An important test for MIS, remote control, and automated advancement is the lack of tactile measurements for healthcare providers. Tactile input devices will greatly support the adoption of such designs. It can be used for both remote control and collaborating devices to relieve the burden of clinical professionals who materialize very fragile frameworks or violate security restrictions.

The article "Clinical Application of Augmented Reality in Computerized Skull Base Surgery" was retracted in 2023. Reasons: unreliable results or conclusions; concerns about the data; concerns about the peer review; concerns about the citations.

At this stage, it has been found that AR is not best at providing meticulous accuracy and guidance, but further limits the duration of activity [44]. However, due to the multifaceted nature of the AR architecture, the total duration of the medical procedure is usually multiplied by the preoperative strategy. Upgrading the mechanized skull can limit the entire season of close interaction. Further consideration should be given to the improvement of the displacement device strategy including design separation and guidance devices to ensure ergonomics and accuracy. Also, a qualified PC is essential for accurate image reproduction. Progress is needed to improve and computerize recreation strategies. Continuous clinical imaging equipment can also make a difference. An ideal basis for sophisticated augmented reality would include no or fewer alignment techniques and no external anchor edges and global positioning structures. However, at this point, it seems that the prudent negotiation process should be stopped early rather than prudent measures. In addition, all devices must be properly coordinated with environmental factors for smooth operation. The ability to subjectively convey the uniqueness of a chosen interaction and the ability to quickly log back in can be one of the important benefits of AR innovation. Pre-programmed warning systems that rely on scores can similarly play a key role in ensuring the safety of managers. In most cases, steady movement is required, as transport and elegance have a huge impact on creating the right design. The throughput rates made for the AR framework range from 5 to 40 edges depending on 2d (fps). More fps requires caution, but the limit of installed frameworks is around 10 frames per second. Running on a GPU significantly increases processing time, producing up to 60 frames per second [9, 78]. To decipher persistent blurry visual results, experts must point to the most uncontrollable rate of 17 frames per second [84]. With these issues in mind, you can carefully construct different queries for useful systems in AR.

1. Ease of implementation and preparation before use
2. Minimum calibration procedure
3. A general interest in virtual objects and photographs in the real world
4. Qualitative (sub-millimetric for science)
5. Minimum registration period
6. Single fusion of surgical equipment
7. Reduced burden
8. Depth indication of both virtual objects and devices
9. Overlay virtual objects only when needed
10. HD resolution and high frame rate
11. Minimum latency
12. Adaptable appropriate contrast of the target image throughout the projection

A new investigation of endoscopic-based skull treatment therapy has been demonstrated that the impact of augmented reality structures on the result depends on the working revel of the specialist [44]: Although augmented reality ordinarily saves careful time and mental exertion, the level of advancement relates to the absence of involvement of the clinical master. Augmented reality constructions might help the presentation of specialists with helpless abilities close to the degree of reasonably capable specialists. The expanded technicity of the greatest gadgets needs special information to be effectively utilized. This likewise plays a critical capacity in acknowledgment of such constructions since the potential impacts of wrong use may be broad. Further in-force examinations ought to be embraced to demonstrate the predominance and advantage of AR careful frameworks as opposed to ordinary strategies. Aside from expanding careful revel in, AR might help instruction by applying rethinking careful preparing and educating methods.

The article "Clinical Application of Augmented Reality in Computerized Skull Base Surgery" was retracted in 2023. Reasons: unreliable results or conclusions; concerns about the data; concerns about the peer review; concerns about the citations.

Natural outlines may be proposed to students giving an all the more full and far-reaching clarification of the life structures and running statute of each organ. As per a new survey, 81% of undergrads energized the consolidation of any such device into their residency programming albeit 93% allowed its usage inside the activity room [54].

Artificial intelligence-based augmented reality has been applied for providing support to investigation and ID in other important disciplines. The most exactness got is 84% that is superior to uninformed specialists (45%) all things considered more awful than master specialists (95%) related to a new glance at [85, 86]. Progressed engineered insight approaches have never longer been applied fittingly inside the cerebral base district since those calculations are very delicate to instruction data, and the accuracy of existing calculations is not adequately correct to be carried out in this space. Right now, such situations are handiest being applied in submit handling of logical snap pictures, which do not now incur quick risk to patients (to order or area-positive designs) (to arrange or portion-positive constructions). This suggests the need of updating the robotized PC creative and farsighted calculations sooner than they might be done in real-time careful applications. Presentation of AR innovation in careful robot frameworks may maybe incredibly support the usefulness of such constructions. New qualities in miniature and nanorobots and independent careful frameworks might be particularly worthwhile.

## 7. Conclusion

Augmented reality is a solid device, which has a possibility to change the cranial-based careful treatment through expanding the careful experience and giving additional data in a protected, easy-to-use, and instinctive strategy. Late examinations show that route structures fusing AR convey comparable outcomes to standard route structures as far as exactness with better ergonomics and AR has been utilized in a few parts of the functional control such as forecast, medical procedure preplanning, navigational, intraoperative imaging, and MIS strategies. AR furthermore might be powerful for instructing capacities. In any case, extra exertion actually must be led to expand the state-of-the-art country, gain the most extreme insurance and trustworthiness, and diminish machine cost. Recent fads in advanced mechanics, representation, area sensors, haptics, engineered insight, and PC innovative and farsighted methods may all help the AR age in its large acknowledgment among specialists. Even though AR provides an efficient way to visualize the cranial base surgery, it is not possible to interact with visualize objects so in future integration of both augmented reality and virtual reality (VR) can be used to interact with visualize objects of cranial base surgery.

## Figures and Tables

**Figure 1:** Correlation between the designs of normal route framework (a) and a route framework coordinating AR (B) (b). GPU: graphic processing unit.

**Figure 2:** Projection of cranial region and cranial nerves.

**Figure 3:** Technical requirements of AR-based general cranial base practices.

**Figure 4:** Technical requirements of AR-based minimally invasive cranial base methods.

**Figure 5:** Augmented reality endoscopic-based skull surgical technique with an enlarged field of view [27].

**Figure 6:** AR display with picture overlay example.

**Figure 7:** Image of AR show with navigation aids depicting anterior sinus outflow [4].

The article "Clinical Application of Augmented Reality in Computerized Skull Base Surgery" was retracted in 2023. Reasons: unreliable results or conclusions; concerns about the data; concerns about the peer review; concerns about the citations.

## Data Availability

The data used to support the findings of this study are included in the article. Should further data or information be required, these are available from the corresponding author upon request.
